The article "Rhodomyrtus tomentosa (Aiton) Hassk. (haramonting) protects against allethrin-exposed pulmo damage in rats: mechanistic interleukins" was retracted in 2026. Reasons: duplicated images; unreliable data; unreliable results or conclusions.

# *Rhodomyrtus tomentosa (Aiton) Hassk.* (haramonting) protects against allethrin-exposed pulmo damage in rats: mechanistic interleukins

**DOI:** 10.3389/fphar.2024.1343936

**Published:** 2024-02-06

**Authors:** Putri Cahaya Situmorang, Syafruddin Ilyas, Rony Abdi Syahputra, Alexander Patera Nugraha, Mimmy Sari Syah Putri, Cheryl Grace Pratiwi Rumahorbo

**Affiliations:** ^1^ Study Program of Biology, Faculty of Mathematics and Natural Sciences, Universitas Sumatera Utara, Medan, Indonesia; ^2^ Department of Pharmacology, Faculty of Pharmacy, Universitas Sumatera Utara, Medan, Indonesia; ^3^ Department of Orthodontics, Faculty of Dental Medicine, Universitas Airlangga, Surabaya, Indonesia; ^4^ Study Program of Mathematics, Faculty of Mathematics and Natural Sciences, Universitas Sumatera Utara, Medan, Indonesia

**Keywords:** IL-1β, IL-6, IL-8, IL-9, IL-10, IL-18

## Abstract

Inhaling Allethrin (C19H26O3) may induce oxidative stress in lung cells by causing the formation of free radi-cals. Interleukins (IL) are a group of secreted cytokines or proteins and signaling molecules initially produced as an immune response by leukocytes. *Rhodomyrtus tomentosa (Aiton) Hassk.* (haramonting) contains antioxidants that may prevent lung damage induced by allethrin-containing electric mosquito repellents. In this study, six groups of rats were exposed to allethrin via an electric mosquito repellent, including positive, negative, and comparison control groups and three groups were administered Rhodomyrtus tomentosa (Aiton) Hassk at 100 mg/kg BW, 200 mg/kg BW, and 300 mg/kg BW. After 30 days, the pulmonary tissue and the blood were taken for immunohisto-chemical and ELISA analysis. The accumulation of inflammatory cells causes the thickening of the alveolar wall structures. Injuries were more prevalent in the A+ group than in the other groups. The connection between the alveoli and blood capillaries, which can interfere with alveolar gas exchange, is not regulated, and the lu-minal morphology is aberrant, causing damage to the alveolar epithelial cells. Exposure to electric mosquito coils containing allethrin can increase the expression of interleukin-1, interleukin-8, interleukin-9, and interleu-kin-18 in blood serum and tissues while decreasing the expression of interleukin-6 and interleukin-10. Like the Vitamin C group, Rhodomyrtus tomentosa can increase alveolar histological alterations by decreasing the ex-pression of IL-1β, IL-8, IL-9, and IL-18 while increasing IL-6 and IL-10. So that this plant can be developed in the future as a drug to prevent lung harm from exposure.

## 1 Introduction

Technological advancements are advancing rapidly with the evolution of mosquito-repellent products. One of them is an electric form that does not produce smoke, such as mosquito coils, which has piqued the interest of many people, or people believe electric mosquito repellents are safer and more effective (Enayati et al., 2007). In Indonesia, mosquitoes are viewed as a vector for various diseases; consequently, many Indonesians use mosquito repellents, including electric mosquito repellent, to prevent mosquito bites (Ipa et al., 2020). First, however, we must be aware that Allethrin (C19H26O3) is a compound derived from pyrethroids that are used in electric mosquito repellents to eradicate mosquitoes and other insects that risk human health (Gargouri et al., 2018). The accumulation of allethrin in the body can form free radicals that induce oxidative stress in cells, a precursor to cancer (Arif et al., 2021). Through the production of free radicals, allethrin induces toxicity via oxidative stress. Hydrogen peroxide is a type of dangerous free radical (Gargouri et al., 2018). The toxic metabolism of the organism produces hydrogen peroxide. Hydrogen peroxide can generate harmful hydroxyl radicals through the Fenton and Haber-Weiss reactions (Phaniendra et al., 2015). Due to exposure to various free radicals, living organisms develop various defense mechanisms, including catalase, an enzymatic antioxidant defense (Phaniendra et al., 2015). If the insect repellent is inhaled or ingested for an extended period, serious side effects may occur (Naz et al., 2019). When used routinely, the active ingredients in electric mosquito repellents can gradually affect and cause abnormalities in the lungs and other organs of the human body (Naz et al., 2019).

The article "Rhodomyrtus tomentosa (Aiton) Hassk. (haramonting) protects against allethrin-exposed pulmo damage in rats: mechanistic interleukins" was retracted in 2026. Reasons: duplicated images; unreliable data; unreliable results or conclusions.

The lungs are susceptible to interference as an organ of the body interacting with the outside world. As a consequence of exposure to hazardous particles, the structure of the lungs is disturbed and damaged (Neves et al., 2019). After exposure to mosquito repellents, alterations in the weight and color of the lungs of rats provide evidence of this disturbance (Hazarika et al., 2022). According to research, long-term use of mosquito repellents containing allethrin may increase the potential of developing ARI (Hazarika et al., 2022). Aside from a high temperature, dizziness, and shortness of breath, this illness can cause a cough, a runny nose, nasal congestion, a sore throat, lethargy, and vertigo (Neves et al., 2019). In addition, molecular studies show that allethrin activates the PI3K/AKT/mTOR messaging pathway, leading to oxidative damage, apoptosis, and autophagy (Jalouli et al., 2022).

Leukocytes produce a cytokine class called interleukins (IL) (Kany et al., 2019). Interleukins regulate cell growth, differentiation, and activation across immune and inflammatory responses (Kany et al., 2019). Interleukins are a protein superfamily that can cause a variety of responses in tissue and cell by binding to specific high-affinity cell surface receptors (Dinarello, 2018). Physical activity is one of the most effective mechanisms for lowering pro-inflammatory interleukin production because it strengthens the immune system (Taherkhani et al., 2020). Other processes that may affect the fat tissue include tissue inflammation decrease and, ultimately, the correction of hypoxia (Taherkhani et al., 2020).

The article "Rhodomyrtus tomentosa (Aiton) Hassk. (haramonting) protects against allethrin-exposed pulmo damage in rats: mechanistic interleukins" was retracted in 2026. Reasons: duplicated images; unreliable data; unreliable results or conclusions.

The cytokine family IL-1 comprises 11 members; the lung is one of many essential tissues mediating fibrosis and inflammatory conditions (Borthwick, 2016). Seven of these members serve as agonists, the remaining three act as receptor antagonists, and the remaining member is an anti-inflammatory cytokine (Taherkhani et al., 2020). IL-1 is a vital inflammatory mediator (Borthwick, 2016). While it is essential to the body’s ability to fight off infection, chronic sickness and acute injury contribute to tissue damage. IL-6 contributes vital functions in inflammatory conditions, immunology, and hematopoiesis and promotes fibrosis formation (Borthwick, 2016). IL-6 is widely acknowledged as a crucial actor in host defense due to its several roles in the immunological and hematopoietic function and causing an acute phase response (Tanaka et al., 2014). One of the most critical functions of IL-8 is inflammation, which helps bring more immune cells, like neutrophils, to infected areas (Cesta et al., 2022). Epithelial cells, which are smooth muscle cells in the respiratory system, also emit IL-8 in addition to macrophages (Cesta et al., 2022). Some of the impacts of IL-8 signaling include increased cancer cell, endothelial cell, and myeloid-derived suppressor cell motility (Pease and Sabroe, 2002). Inflammation with eosinophils, Hyperplasia, and hypertrophy of the mucosal vessels, as well as hyperresponsiveness of the bronchial tubes, are just some of the physiological changes within the respiratory tract that have been related to the pleiotropic cytokine IL-9 (Li et al., 2022). IL-10 is a cytokine that functions as an anti-inflammatory that aids in regulating the body’s defenses to diseases, thereby protecting the organism from infection and maintaining tissue homeostasis (Iyer and Cheng, 2012). IFN production is another inflammatory cytokine that IL-18 greatly stimulates. Macrophages, dendritic cells, lymphocytes, and even specific nonimmune cells may produce IL-18 (Ihim et al., 2022).

*Rhodomyrtus tomentosa (Aiton) Hassk.*, or haramonting, is a typical North Sumatera herbal plant containing acyl phloroglucinol, flavonoids, tannins, Rhodomyrtone, and acyl phloroglucinol (Zhang et al., 2018; Situmorang et al., 2022). This plant has been shown to enhance the histology of the testicles, liver, and cervical cancer (Irianti et al., 2020; Situmorang et al., 2023). This investigation examines the expression of the interleukin family in rat lung tissue and blood serum following exposure to allethrin via electric mosquito repellent. It is anticipated that the high antioxidant content of R. tomentosa can eventually be turned into herbal medicine, particularly for preventing lung damage caused by allethrin-containing electric mosquito repellents.

The article "Rhodomyrtus tomentosa (Aiton) Hassk. (haramonting) protects against allethrin-exposed pulmo damage in rats: mechanistic interleukins" was retracted in 2026. Reasons: duplicated images; unreliable data; unreliable results or conclusions.

## 2 Materials and methods

### 2.1 Chemical and reagents

The antibodies used for the ELISA kit were ELISA Kit IL-1β PitokineR (Catalog number: EKO393-CAP), ELISA Kit Rat IL-6 (Catalog#E-E1-R0015, Elabscience), Rat IL-8 CXCL8 Elisa Kit (Catalog#Abx576575, Abbexa). Rat IL-9 ELISA Kit (Catalog#ERA34RB, ThermoFisher, United States), Rat IL-10 ELISA Kit (Catalog#ab214566, Abcam, United States) and Rat IL-18 ELISA Kit (Catalog#ab213909, Abcam, United States). The antibodies used for Immunohistochemistry were Invitrogen IL-1β Polyclonal Antibody (Catalog #PA5-119221,ThermoFisher Scientific, United States), Invitrogen IL-6 Monoclonal Antibody (Catalog #AHC0762, ThermoFisher Scientific, United States), Invitrogen IL-8 (CXCL8) Polyclonal Antibody (Catalog # PA5-79113, ThermoFisher Scientific, United States), Bios IL-9 Polyclonal Antibody (Catalog#BS-2428R,ThermoFisher, United States), Invitrogen IL-10 Polyclonal Antibody (Catalog# PA5-94918, ThermoFisher Scientific, United States), Invitrogen IL-18 Polyclonal antibody (Catalog#PA5-79481, ThermoFisher Scientific, United States). Storage buffer solution (Catalogue # BS-0812R) was phosphate buffer solution (PBS) containing 50% glycerol and 1% bovine serum albumin (BSA).

### 2.2 Preparation of the *Rhodomyrtus tomentosa*

*Rhodomyrtus tomentosa (Aiton) Hassk* (Myrtaceae family) Leaves are mostly cultivated in the Berastasi region of Sumatera Utara Province, Indonesia. Registration number 012/MEDA/2022 at the Medanense Botanical Herbarium indicates that Dr. Nursahara Pasaribu, MSc of Universitas Sumatera Utara identified and approved the voucher in Medan, Indonesia. Afterwards, the object is subjected to a purification procedure that includes washing and subsequent natural drying. A quantity of 1.02 kg of *R. tomentosa (Aiton) Hassk* leaf powder was extracted by maceration in technical ethanol (70%) until fully submerged. The solvent used for extraction was replaced every 24 h. Upon acquiring an ethanol extract, it was subjected to evaporation in order to produce a concentrated ethanol extract. The formulation of this recipe was optimized for the oil phase, surfactants, and co-surfactants. A 0.5 mg dosage of *R. tomentosa (Aiton) Hassk* extract was added to the Tween 20 solution for sonification. Prior to the addition of capriol 90 and homogenization, PEG 400 was introduced and subjected to sonication. The resulting product is diluted at a ratio of 1 part product to 100 parts distilled water, and then thoroughly mixed using an ultrasonic equipment to ensure uniformity (Ilyas et al., 2021).

The article "Rhodomyrtus tomentosa (Aiton) Hassk. (haramonting) protects against allethrin-exposed pulmo damage in rats: mechanistic interleukins" was retracted in 2026. Reasons: duplicated images; unreliable data; unreliable results or conclusions.

### 2.3 Animal handling

This investigation utilized 36 male of *Rattus norvegicus.* Male rats are 180–200 g in weight and 10–14 weeks old. Each group of six male rats contained six male rats was divided into six groups. Two weeks were used to acclimate male rats to the laboratory environment before they were placed in an enclosure with a constant room temperature (25.0.3°C) and humidity level (35%–60%). The cage was illuminated for 12 h, followed by 12 h of darkness. Male Rats were fed corn and pellets *ad libitum* and had unrestricted access to water. Rats were placed in a 40 cm × 30 cm plastic container. The rodents were placed in a 40-by-30-cm plastic case. The research was conducted with sanction from the USU FMIPA Medan Health Research Ethics Committee (No. 0896/KEPH-FMIPA/2022).

### 2.4 Research design

These investigations were conducted using a Randomized Complete Design (RCD). This form of study is referred to as an experimental study. One month was spent exposing rats to an electric mosquito repellent containing allethrin. In this investigation, six treatment groups were investigated. A-are negative control, A+ are rat exposed to allethrin, A1 are rat administered 0.2 mg/kg BW of vitamin C and then exposed to allethrin, A2 are rat administered 100 mg/kg BW of *R. tomentosa* and then exposed to allethrin, and A3 are rat administered 200 mg/kg BW of vitamin C and then exposed to allethrin. *Rhodomyrtus tomentosa* was then exposed to allethrin, and A4 were rat that was administered 300 mg/kg BW of *R. tomentosa* that was then exposed to allethrin. Within 30 days, administration of *Rhodomyrtus tomentosus* and exposure to an allethrin-containing mosquito repellent for 3 hours. After 30 days, a ketamine injection was administered for surgery, and the lungs and blood were removed for immunohistochemical and ELISA analysis, respectively.

### 2.5 Measurement of haematology parameters

A sterile pipette was used to obtain blood samples from the heart. To prevent hemolysis, water exposure was avoided. Within a microcentrifuge tube containing 0.5 mL, an anticoagulant solution consisting of 10 mL/1 mL EDTA was added. The City of Medan Health Laboratory ran the hematology tests. According to the guidelines provided by the manufacturer, each sample was analyzed three times.

The article "Rhodomyrtus tomentosa (Aiton) Hassk. (haramonting) protects against allethrin-exposed pulmo damage in rats: mechanistic interleukins" was retracted in 2026. Reasons: duplicated images; unreliable data; unreliable results or conclusions.

### 2.6 Measurement of MDA, NGAL, and SOD

Measurements of MDA, NGAL, and SOD were obtained from blood samples collected from the heart. The duplicate reagent was poured to 50 mL wells, and blood samples were added to the rest. Each well received 50 mL biotinylated detection ab working solution. After covering the plate, 45 min were spent in an incubator at 37°C. After incubation, each well was refilled with 350 mL of wash buffer. The buffer was allowed to sit for a couple of minutes. After drying with absorbent paper, the solution was removed from each well. After three washing, each well received 100 L of HRP conjugate working solution. The dish was covered again and incubated at 37°C for 30 min. Each well received 90 mL substrate reagent following incubation. After that, a new cover plate was placed over everything and incubated at 37°C for 15 min. After the final incubation, each well received 50 mL of stop solution and the plate was covered to prevent light exposure for MDA Analysis. Regarding the measurement of NGAL, Subjected to centrifugation at a speed of 4,230 revolutions per minute for a duration of 5 minutes. After removing the supernatant, the samples were partitioned into three 0.5 cc containers. Prior to the evaluation, the samples were subjected to freezing and stored at a temperature of −200°C. The measurements were conducted using a commercial NGAL. Regarding the measurement of SOD, The standard solution was transferred into microplate wells using Eppendorf tubes. The microplate’s empty wells received 0.1 mL of sample diluent buffer and rat blood serum as controls. The lid was a 90-min microplate replica heated at 37°. The cover was removed and the wells emptied and transferred to tissue paper to remove any liquid from the microplate. Each well received 0.1 mL biotin SOD antibody solution. Reader. After sealing, the microplate was incubated at 37°C for 60 min. Each well received 0.1 mL of streptavidin-biotin complex (SABC) solution after incubation. After that, we covered the microplate and incubated it at 37°C for 30 min 90 L of TMB were pumped into each well after five wash buffer rinses. The microplate was sealed and incubated at 37°C for 25–30 min to turn blue. An ELISA reader at 450 nm measured OD absorbance.

### 2.7 Enzyme-linked immunosorbent assay (ELISA)

The initial blood sample was extracted from the rat’s cardiac organ. To avoid coagulation, the blood should be placed in a tube containing an anticoagulant such as EDTA or citrate. The vials were incubated at ambient temperature for a duration of 10–20 min, followed by centrifugation at a speed of 2000–3,000 revolutions per minute for a period of 20 min. Subsequently, the gathered liquid portion might be utilized for examination. Subsequently, ten-well microplates were employed to create the standards. Dispense 100 μL of standard diluent into well 1 and 50 μL into well 2. Wells 3 and 4 each hold 50 μL of liquid, which is a portion of the total liquid found in wells 1 and 2. Similarly, wells 5 and 6 augment the solution volume by an additional 50 ul compared to the previous well, and this pattern continues until wells 9 and 10, when there is an additional 50 ul compared to the preceding wells. Subsequently, the mixture was incubated for a duration of 30 min at a temperature of 37°C, continuing throughout the night. The washing solution was made by dissolving 1 mL in 29 mL of distilled water. Subsequently, following the depletion of the well, proceed to cleanse it on five occasions using the washing solution prepared in Step 3. To facilitate the attachment of the antigen in the sample to the plate, introduce blocking buffer onto the plate and allow it to incubate for a duration of 60 min at a temperature of either 37°C or 40°C for a period of 24 h. Each well was filled with a 10:40 ratio of sample to diluent, with 10 ul of sample and 40 ul of diluent. Place the piece directly at the lowest point of the well. Next, it is necessary to meticulously blend the sample and sample diluent. Place the plate in a heated incubator and maintain it at a warm temperature for a duration of 120 min. Add 100 µM of biotinylated antibody to each well. The incubation period should last 24 h at a temperature of 37°C, with a duration of 60 min. The well should be emptied and the cleaning solution prepared in Step 3 should be used to cleanse the well on five separate occasions. Add 100 μL of ABC solution into each well. Place in a storage area with a temperature of 370°C for a duration of 30 min. Subsequently, drain the well and vigorously clean it with the washing solution prepared in Step 3 on five occasions. Subsequently, each well was subjected to treatment with 90 ul of HRP conjugate and 90 ul of TMB. Allow the plate to remain at a temperature of 370°C for a duration of 30 min. We introduced 100 μL of stop solution into each well, resulting in a transition from a blue color to a yellow tint. The determination of optical density (OD) values should be conducted using an ELISA reader set at a wavelength of 450 nm, with each sample being replicated three times (Simanullang et al., 2022a; Simanullang et al., 2022b).

The article "Rhodomyrtus tomentosa (Aiton) Hassk. (haramonting) protects against allethrin-exposed pulmo damage in rats: mechanistic interleukins" was retracted in 2026. Reasons: duplicated images; unreliable data; unreliable results or conclusions.

### 2.8 Immunohistochemistry

IL-1β, IL-6, IL-8, IL-9, IL-10, and IL-18 were analyzed by immunohistochemistry to determine the histological effects of Rhodomyrtus tomentosa administration on the expression of several cytokines. The thickness of the paraffin-embedded lung tissue was between 4–5 microns. The tissue was pretreated by being heated at pH 6.0 and 350W in a citrate buffer. Antibodies against IL-1β, IL-6, IL-8, IL-9, IL-10, and IL-18 were incubated with the tissue after a PBS wash. Analysis of IL-1 in paraffin-embedded lung tissue. Polyclonal antibody (Product # PA5-119221) was used at 20 g/mL, and HRP-Linked Caprine Anti-Rabbit IgG was used at 2 g/mL, both in separate incubations with the samples. Overnight incubation at 4°C and 95% humidity with 1:20 dilution of IL-6 monoclonal antibody (Product # AHC0762) in 3% BSA-PBS. Storage buffer PBS containing 5 mg BSA was used to incubate IL-8 (CXCL8) with polyclonal antibody against IL-8 (CXCL8). Peroxidase-conjugated goat anti-rabbit IgG was employed as the secondary antibody, and the incubation temperature was set to 37°C for 30 min. DAB was used as the chromogen in conjunction with the HRP Conjugated Rabbit IgG Super Vision Assay Kit to create an image of the tissue segment. Anti-IL-9 Polyclonal Antibody, Unconjugated (bs-2428R) was used to label formalin-fixed, paraffin-embedded rat lungs at a dilution of 1:200, with a secondary antibody conjugate and DAB staining following. Next, 1 g/mL rabbit anti-IL10 antibody (Product # PA5-94918) was incubated with the tissue segment at 4°C for 24 h. Peroxidase-conjugated goat anti-rabbit IgG was employed as the secondary antibody, and the incubation temperature was set to 37°C for 30 min. Use a 1 g/mL dilution of the polyclonal antibody (Product # PA5-79481) against IL-18 (overnight at 4°C), followed by 30 min at 37°C with biotinylated goat anti-rabbit IgG. Staining with haematoxylin Mayer followed a chromogenic visualisation process with 3,3-diaminobenzidine (DAB) hydrochloride (Ilyas et al., 2022).

### 2.9 Statistical analysis of data

Average and standard deviation figures are provided for the data. The data was analyzed using SPSS 24’s ANOVA and Kruskal–Wallis tests (for non-parametric data).

## 3 Results

### 3.1 Effect of *Rhodomyrtus tomentosa* on hematology parameters of allethrin-exposed rats

Hematological parameters were altered in Rats after treatment of 100–300 mg/kg BW of haramonting, as reported in Table 1. Hematological parameters were substantially different between groups A+ and B after administration of 100 mg/kg BW of haramonting. Hemoglobin, SGOT, and SGPT were substantially different in the Rhodomyrtus tomentosa 200 mg/kg BW group compared to the A+ group. Hemoglobin, leukocytes, lymphocytes, eosinophils, monocytes, SGOT, SGPT, and creatinine were substantially different in the 300 mg/kg BW group compared to the A+ group, but were comparable in the vitamin C or control groups (A1). Neither neutrophils, hematocrit, nor urea differed across groups (*p* > 0.05). The hematological data in Table 1 indicate that administration of 100–300 mg/kg BW of Rhodomyrtus tomentosa has an effect on the hematological parameters of rats, excluding neutrophil, hematocrit, and urea levels. In all categories, neutrophil, hematocrit, and urea levels are considered normal.

The article "Rhodomyrtus tomentosa (Aiton) Hassk. (haramonting) protects against allethrin-exposed pulmo damage in rats: mechanistic interleukins" was retracted in 2026. Reasons: duplicated images; unreliable data; unreliable results or conclusions.

**TABLE 1:** *Effect of Rhodomyrtus tomentosa on Hematology parameters of* allethrin-exposed rats.

Hematology	Unit	Treatments (Mean ± SD)					
		A-	A+	A1	A2	A3	A4
Hemoglobin	g/dL	13.72 ± 0.41	28.07 ± 3.02^#^	15.44 ± 1.02^*^	27.08 ± 2.24	20.11 ± 2.07	16.44 ± 2.92^*^
Erythrocytes	x10^6^/µL	8.51 ± 0.22	9.07 ± 0.06^#^	8.59 ± 0.04	8.69 ± 2.03	8.65 ± 1.04	8.60 ± 0.01
Leukocytes	x 10^3^/µL	8.59 ± 0.23	13.03 ± 0.82^#^	9.02 ± 0.92^*^	12.76 ± 2.22	11.02 ± 1.02	9.32 ± 0.07^*^
Haematocrit	%	43.79 ± 1.03	47.08 ± 2.07	43.70 ± 2.01	46.09 ± 9.13	42.41 ± 4.20	42.70 ± 5.03
Neutrophils	x 10^3^/µL	1.44 ± 0.09	3.04 ± 0.07^#^	1.48 ± 0.02^*^	3.02 ± 0.04	2.91 ± 0.01	1.48 ± 0.02
Lymphocytes	x 10^3^/µL	5.86 ± 0.07	8.81 ± 1.07^#^	5.91 ± 0.34^*^	8.04 ± 1.97	7.22 ± 1.13	5.82 ± 0.04
Eosinophils	x 10^3^/µL	0.048 ± 0.01	0.099 ± 0.01^#^	0.050 ± 0.01^*^	0.082 ± 0.01	0.067 ± 0.01	0.055 ± 0.01^*^
Monocytes	x 10^3^/µL	0.471 ± 0.03	0.872 ± 0.01^#^	0.501 ± 0.01^*^	0.774 ± 0.02	0.603 ± 0.01	0.582 ± 0.01^*^
SGOT	u/L	114. 21 ± 4.81	231.92 ± 8.55^#^	115.07 ± 9.11^*^	200.95 ± 9.78	188.07 ± 9.81*	117.06 ± 9.21^**^
SGPT	u/L	50.16 ± 3.22	162.07 ± 12.09^##^	52.19 ± 10.02^*^	153.25 ± 9.56	86.91 ± 8.77*	55.39 ± 9.92^**^
Creatinine	mg/dL	0.44 ± 0.01	0.78 ± 0.01^#^	0.49 ± 0.02^*^	0.70 ± 0.02	0.61 ± 0.02	0.55 ± 0.01^*^
Ureum	mg/dL	21.09 ± 1.11	38.01 ± 3.22^#^	22.11 ± 3.15^*^	36.24 ± 1.29	32.42 ± 0.96	23.11 ± 2.95^*^

A-: control, A+: allethrin-exposed rats, A1: allethrin-exposed rats +0.02 mg Vitamin C, A2: allethrin-exposed rats +100 mg/Kg BW, of *Rhodomyrtus tomentosa*, A3: allethrin-exposed rats +200 mg/Kg BW, of *Rhodomyrtus tomentosa*, A4: allethrin-exposed rats +300 mg/Kg BW, of *Rhodomyrtus tomentosa*, (^#^ *p* < 0.05 vs A-.

##*p* < 0.01 vs A-, *p < 0.05 compared A+, **p < 0.01 vs A+).

### 3.2 Effect of *Rhodomyrtus tomentosa* of allethrin-exposed rats on level of SOD, MDA and NGAL

When compared to groups A- and A1, there were significant differences found in the levels of SOD, MDA, and NGAL in rodents that had been exposed to allethrin (*p* < 0.05 or *p* = 0.030). The SOD levels of rats given 100 or 200 mg/kg BW of *R. tomentosa* were significantly different from those of rats in the A+ group, with the difference decreasing with higher dosages of these botanicals. *Rhodomyrtus tomentosa* reduced MDA levels compared to the A+ group at a dosage of 300 mg/kg BW (Table 2). *Rhodomyrtus tomentosa* reduced levels of MDA and NGAL in a dose-dependent manner. Antioxidants found in *R. tomentosa* have been shown to increase SOD activity and decrease serum levels of MDA and NGAL. *Rhodomyrtus tomentosa* has been shown to increase SOD activity, which in turn protects cells against oxidant disturbances and oxidative stress, both of which can lead to a number of lung disorders and injuries. Increased MDA and NGAL levels, along with reduced SOD activity, are indicators of increased lipid peroxide caused by an antioxidant deficiency.

The article "Rhodomyrtus tomentosa (Aiton) Hassk. (haramonting) protects against allethrin-exposed pulmo damage in rats: mechanistic interleukins" was retracted in 2026. Reasons: duplicated images; unreliable data; unreliable results or conclusions.

**TABLE 2:** Effect of *Rhodomyrtus tomentosa of* allethrin-exposed rats on level of SOD, MDA and NGAL.

Parameters	Unit	Groups (Mean ± SD)					
		A-	A+	A1	A2	A3	A4
SOD	pg/mL	23.88 ± 2.41	14.62 ± 1.69^#^	23.21 ± 3.02*	18.12 ± 2.04	20.88 ± 0.09*	23.91 ± 3.04*
MDA	µM/L	8.45 ± 0.03	12.87 ± 2.88^#^	8.40 ± 1.09*	10.34 ± 2.21	9.87 ± 1.03*	8.81 ± 1.03*
NGAL	Ng/mL	0.215 ± 0.01	0.667 ± 0.01^#^	0.212 ± 0.01*	0.581 ± 0.01	0.435 ± 0.01*	0.235 ± 0.01*

A-: control, A+: allethrin-exposed rats, A1: allethrin-exposed rats +0.02 mg Vitamin C, A2: allethrin-exposed rats +100 mg/Kg BW, of *Rhodomyrtus tomentosa*, A3: allethrin-exposed rats +200 mg/Kg BW, of *Rhodomyrtus tomentosa*, A4: allethrin-exposed rats +300 mg/Kg BW, of *Rhodomyrtus tomentosa*, (^#^ *p* < 0.05 vs C-, *p < 0.05 vs C+).

### 3.3 Morphological and histological analysis of the lungs of allethrin-exposed rats after administration of *Rhodomyrtus tomentosa*

The color of the lungs differed between the control group (A-) and the allethrin exposure group (A+), with A-exhibiting a rich red hue and A+ exhibiting a pale hue with spots around the organs. Spots were also observed following administration of haramonting, but they diminished as the dose was increased (Figure 1). Rats exposed to an electric mosquito repellent containing allethrin developed lung injury. Based on histological findings (Figure 2), both Group A- (control) and Group A1 had thickened alveolar membranes, but lumen size and alveolar density varied. However, herbal administration (A2 to A4) elongated the alveolar connections, diminished the cell nucleus, and weakened the cell membrane. The accumulation of inflammatory cells in the alveolar wall structures led to their thickening. The incidence of injury was greater in the A+ group than in the other groups. Damage is also observed in the alveolar epithelial cells as a result of the connection between the alveoli and blood capillaries, in which the alveolar gas exchange is not tightly regulated and the lumen morphology is irregular.

The article "Rhodomyrtus tomentosa (Aiton) Hassk. (haramonting) protects against allethrin-exposed pulmo damage in rats: mechanistic interleukins" was retracted in 2026. Reasons: duplicated images; unreliable data; unreliable results or conclusions.

**FIGURE 1:** The lung Morphological of allethrin-exposed rats after administration of *Rhodomyrtus tomentosa.* **(A-)**: Control, **(A+)**: allethrin-exposed rats, **(A1)**: allethrin-exposed rats +0.02 mg Vitamin C, **(A2)**: allethrin-exposed rats +100 mg/Kg BW of *Rhodomyrtus tomentosa*, **(A3)**: allethrin-exposed rats +200 mg/Kg BW of *Rhodomyrtus tomentosa*, **(A4)**: allethrin-exposed rats +300 mg/Kg BW of *Rhodomyrtus tomentosa.*

**FIGURE 2:** Histological analysis of the lungs of allethrin-exposed rats after administration of *Rhodomyrtus tomentosa.* **(A-)**: Control, **(A+)**: allethrin-exposed rats, **(A1)**: allethrin-exposed rats +0.02 mg Vitamin C, **(A2)**: allethrin-exposed rats +100 mg/Kg BW of *Rhodomyrtus tomentosa*, **(A3)**: allethrin-exposed rats +200 mg/Kg BW of *Rhodomyrtus tomentosa*, **(A4)**: allethrin-exposed rats +300 mg/Kg BW of *Rhodomyrtus tomentosa.* **(a)**. Membrane, **(b)**. Lumen (40x).

### 3.4 Expression of IL-1β on lung histological changes and serum after administration of *Rhodomyrtus tomentosa* in allethrin-exposed rats

Blood serum from rats was analyzed to determine IL-1β expression. Following the administration of haramonting (*R. tomentosa*) at the lowest dose, rat blood that had been exposed to allethrin via an electric mosquito repellent exhibited a high level of IL-1β expression. *Rhodomyrtus tomentosa* inhibited IL-1 *β* expression noticeably at 200 and 300 mg/kgBW. There is evidence that the highest dose of this plant can inhibit IL-1β production (Figure 3). Kruskal–Wallis tests performed on the nonparametric data showed that there were significant variations in IL-1β expression between the groups (Supplementary Table S3). The Mann-Whitney test showed that there was a statistically significant difference between the A+ group and IL-1β expression (*p* < 0.01, *p* = 0.001). *Rhodomyrtus tomentosa* (100 mg/kg BW) and A2 (100 mg/kg BW) were both below the threshold for statistical significance required to detect a difference. There were no statistically significant changes (*p* > 0.01) between the A+ and control groups at 100 mg/kg BW, but there were at 200 and 300 mg/kg BW. The analysis results in the table are supported by histological changes in the lung tissue due to IL-1β expression. The expression of IL-1 was highest in Group A+ and lowest in Group A- and *Rhodomyrtus* tomentosa at 300 mg/kg BW (Figure 4).

**FIGURE 3:** Expression of interleukins family after administration of *Rhodomyrtus tomentosa* in allethrin-exposed rats. A-: Control, A+: allethrin-exposed rats, A1: allethrin-exposed rats +0.02 mg Vitamin C, A2: allethrin-exposed rats +100 mg/Kg BW of *Rhodomyrtus tomentosa*, A3: allethrin-exposed rats +200 mg/Kg BW of *Rhodomyrtus tomentosa*, A4: allethrin-exposed rats +300 mg/Kg BW of *Rhodomyrtus tomentosa* (^ns^p >0.05, ^##^ *p* < 0.01 vs A-, *p < 0.05 vs A+, **p < 0.01 vs A+).

The article "Rhodomyrtus tomentosa (Aiton) Hassk. (haramonting) protects against allethrin-exposed pulmo damage in rats: mechanistic interleukins" was retracted in 2026. Reasons: duplicated images; unreliable data; unreliable results or conclusions.

**FIGURE 4:** Expression of IL-1β on lung histological changes after administration of *Rhodomyrtus tomentosa* in allethrin-exposed rats. **(A-)**: Control, **(A+)**: allethrin-exposed rats, **(A1)**: allethrin-exposed rats +0.02 mg Vitamin C, **(A2)**: allethrin-exposed rats +100 mg/Kg BW of *Rhodomyrtus tomentosa*, **(A3)**: allethrin-exposed rats +200 mg/Kg BW of *Rhodomyrtus tomentosa*, **(A4)**: allethrin-exposed rats +300 mg/Kg BW of *Rhodomyrtus tomentosa* (^ns^p >0.05, ^##^ *p* < 0.01 vs A-, *p < 0.05 vs A+, **p < 0.01 vs A+).

### 3.5 Expression of IL-6 on lung histological changes and serum after administration *of Rhodomyrtus tomentosa* in allethrin-exposed rats

The comparison group (A1) expressed the most IL-6, followed by the Vitamin C-treated group (A1) and the control group (A-). Allethrin exposure via electric mosquito repellent can reduce IL-6 (A+) expression. Even at the lowest dose, *R. tomentosa* suppressed the production of this protein (A1). The expression of IL-6 was upregulated at 200 and 300 mg/kgBW, although the mean value was the same as in the vitamin C group (Figure 3). The IL-6 expression levels were substantially different between the groups (*p* < 0.01). Expression levels of IL-6 were found to be significantly different between the A group and the A+ group using the Mann-Whitney test (*p* < 0.00, *p* = 0.002). While there was no statistically significant difference between 100 and 300 mg/kg BW of *R. tomentosa,* histological analysis of alterations in this protein (Figure 5) showed that there was an overall decrease. Expression of IL-6 was highest in the A- and A1 groups (control and vitamin C, respectively), and lowest in the A4 group.

**FIGURE 5:** Expression of IL-6 on lung histological changes after administration of *Rhodomyrtus tomentosa* in allethrin-exposed rats. **(A-)**: Control, **(A+)**: allethrin-exposed rats, **(A1)**: allethrin-exposed rats +0.02 mg Vitamin C, **(A2)**: allethrin-exposed rats +100 mg/Kg BW of *Rhodomyrtus tomentosa*, **(A3)**: allethrin-exposed rats +200 mg/Kg BW of *Rhodomyrtus tomentosa*, **(A4)**: allethrin-exposed rats +300 mg/Kg BW of *Rhodomyrtus tomentosa*.

### 3.6 Expression of IL-8 on lung histological changes and serum after administration of *Rhodomyrtus tomentosa* in allethrin-exposed rats

Figure 3 depicts the expression of IL-8 in the blood serum of rats exposed to electric mosquito repellents. When this plant was given at a dose of 100 mg/kg BW, there was no discernible change in IL-8 expression. There was a statistically significant reduction in IL-8 expression at dosages of 200 mg/kg BW (*p* < 0.05) and 300 mg/kg BW (A3). According to the results of the Kruskal–Wallis test presented, there is a statistically significant distinction in IL-8 expression between the groups. According to the Mann-Whitney test, there was a statistically significant difference between the A+ group and the IL-8 expression group (*p* < 0.01, *p* = 0.002). There was insufficient data to determine whether or not *R. tomentosa* (100 mg/kg BW) or A2 (100 mg/kg BW) had any effect. At lower doses (200 and 300 mg/kg BW), there were no statistically significant differences (*p* > 0.05) between the A+ group and the comparator groups (A1 and A-). This can be seen in (Figure 6) The *R. tomentosa* at 300 mg/kg BW (A4) group had the lowest levels of IL-8 expression, followed by group A+ and group A-.

The article "Rhodomyrtus tomentosa (Aiton) Hassk. (haramonting) protects against allethrin-exposed pulmo damage in rats: mechanistic interleukins" was retracted in 2026. Reasons: duplicated images; unreliable data; unreliable results or conclusions.

**FIGURE 6:** Expression of IL-8 on lung histological changes after administration of *Rhodomyrtus tomentosa* in allethrin-exposed rats. **(A-)**: Control, **(A+)**: allethrin-exposed rats, **(A1)**: allethrin-exposed rats +0.02 mg Vitamin C, **(A2)**: allethrin-exposed rats +100 mg/Kg BW of *Rhodomyrtus tomentosa*, **(A3)**: allethrin-exposed rats +200 mg/Kg BW of *Rhodomyrtus tomentosa*, **(A4)**: allethrin-exposed rats +300 mg/Kg BW of *Rhodomyrtus tomentosa* (^ns^p >0.05, ^##^ *p* < 0.01 vs A-, *p < 0.05 vs A+, **p < 0.01 vs A+).

### 3.7 Expression of IL-9 on lung histological changes and serum after administration of *Rhodomyrtus tomentosa* in allethrin-exposed rats

Expression of IL-9 in the blood serum of rats exposed to electric mosquito repellents revealed an increase in IL-9 expression that was not significantly different at 100 mg/kg BW (A2) and 200 mg/kg BW (A3). At the greatest dose, 300 mg/kgBW (A3), there was a significant reduction in IL-8 expression. According to the results of the Kruskal–Wallis test presented in Supplementary Table S1, there is a statistically significant difference in IL-9 expression between the groups. The Mann-Whitney test revealed a statistically significant disparity between the A+ group and the IL-9 expression group (*p* < 0.01, *p* = 0.003). *Rhodomyrtus tomentosa* doses between 100 and 200 mg/kg body weight showed no statistically significant difference (*p* > 0.05) between groups A+. However, when compared to the A+ group, substantial differences emerged at 300 mg/kg BW. The expression of IL-9 was highest in group A+ and lowest in group A- and Vitamin C (A1) (Figure 7). Nevertheless, the administration of this plant yields identical outcomes to those of Vitamin C, so enhancing lung histology, but the histological architecture of the lungs in the untreated group of rats exhibited damage characterized by the initial loss of the alveolar septum, together with the presence of inflammatory cell infiltration and edema, as a result of chemical exposure.

The article "Rhodomyrtus tomentosa (Aiton) Hassk. (haramonting) protects against allethrin-exposed pulmo damage in rats: mechanistic interleukins" was retracted in 2026. Reasons: duplicated images; unreliable data; unreliable results or conclusions.

**FIGURE 7:** Expression of IL-9 on lung histological changes after administration of *Rhodomyrtus tomentosa* in allethrin-exposed rats. **(A-)**: Control, **(A+)**: allethrin-exposed rats, **(A1)**: allethrin-exposed rats +0.02 mg Vitamin C, **(A2)**: allethrin-exposed rats +100 mg/Kg BW of *Rhodomyrtus tomentosa*, **(A3)**: allethrin-exposed rats +200 mg/Kg BW of *Rhodomyrtus tomentosa*, **(A4)**: allethrin-exposed rats +300 mg/Kg BW of *Rhodomyrtus tomentosa* (^ns^p >0.05, ^##^ *p* < 0.01 vs A-, *p < 0.05 vs A+, **p < 0.01 vs A+).

### 3.8 Expression of IL-10 on lung histological changes and serum after administration of *Rhodomyrtus tomentosa* in allethrin-exposed rats

The expression of IL-10 was also evaluated in the blood serum of rats allethrin exposed to electric mosquitoes, which revealed a decrease in IL-10 expression that was not substantially different at 100 mg/kg BW (A2) and 200 mg/kg BW (A3). Figure 3 displayed considerable increase in IL-10 expression at the highest doses of vitamin C (A1) and 300 mg/kgBW (A3). IL-10 expression differed significantly (*p* < 0.01, Supplementary Table S1) between the groups. The Mann-Whitney *U* test revealed a statistically significant difference in IL-10 expression between the A+ group and the other groups (*p* < 0.00, *p* = 0.001). At 100 mg/kg BW of *R. tomentosa*, this difference was not statistically significant. There was a big discrepancy between the A+ dose and the standard dose of 200–300 mg/kgBW. Figure 8 shows that IL-10 expression was highest in the control (A-) and vitamin C (A1) groups and lowest in the A+ group. Histologically, In the untreated group of rats, the alveoli were coated with macrophages. An increase in the number of alveoli can be observed, along with an increase in the number of macrophages or dust cells around the alveoli. The alveoli exhibit a granular texture and seem smooth on the alveolar macrophages. The cytoplasm, which has an oval form, is visible across the whole field of vision. Moreover, alterations in the structure of the membrane. The alveoli become apparent due to the loss of endothelial cells that line the blood vessels around them. This leads to the enlargement of the blood vessels, allowing the blood cells to exit and disseminate. Pulmonary edema is characterized by the swelling of the alveolar surface and widening of the lumen of the alveoli, which can be observed visually. This leads to pulmonary harm and impairs the functioning of the respiratory system. Nevertheless, the administration of this plant yields identical outcomes to those of Vitamin C, so enhancing lung histology.

The article "Rhodomyrtus tomentosa (Aiton) Hassk. (haramonting) protects against allethrin-exposed pulmo damage in rats: mechanistic interleukins" was retracted in 2026. Reasons: duplicated images; unreliable data; unreliable results or conclusions.

**FIGURE 8:** Expression of IL-9 on lung histological changes after administration of *Rhodomyrtus tomentosa* in allethrin-exposed rats. **(A-)**: Control, **(A+)**: allethrin-exposed rats, **(A1)**: allethrin-exposed rats +0.02 mg Vitamin C, **(A2)**: allethrin-exposed rats +100 mg/Kg BW of *Rhodomyrtus tomentosa*, **(A3)**: allethrin-exposed rats +200 mg/Kg BW of *Rhodomyrtus tomentosa*, **(A4)**: allethrin-exposed rats +300 mg/Kg BW of *Rhodomyrtus tomentosa* (^ns^p >0.05, ^##^ *p* < 0.01 vs A-, *p < 0.05 vs A+, **p < 0.01 vs A+).

### 3.9 Expression of IL-18 on lung histological changes and serum after administration of *Rhodomyrtus tomentosa in* allethrin-exposed rats

IL-18 expression was also evaluated in the blood serum of rats exposed to alltehrin from electric mosquitoes, which showed a decrease in expression at each dose level where IL-18 expression was lowest at A-, A1 and followed by the highest dose of *R. tomentosa*, namely, 300 mg/kg BW (A3). Kruskal–Wallis test results (Supplementary Table S1) reveal that there is a statistically significant difference in IL-18 expression across groups. Using the Mann-Whitney *U* test, we found that A+ and B+ groups substantially differed from one another in IL-18 expression (*p* < 0.01, *p* = 0.002). There was no statistically significant difference between *R. tomentosa* (100 mg/kg) and A2 (*p* > 0.02). Histologically Nonetheless, alterations appeared at 200 and 300 mg/kg BW (*p* < 0.05) in Figure 9 when compared to the A+ group. Group A+ showed the highest IL-18 expression, whereas groups A- and *R. tomentosa* 300 mg/kg BW (A4) showed the lowest.

**FIGURE 9:** Expression of IL-18 on lung histological changes after administration of *Rhodomyrtus tomentosa* in allethrin-exposed rats. **(A-)**: Control, **(A+)**: allethrin-exposed rats, **(A1)**: allethrin-exposed rats +0.02 mg Vitamin C, **(A2)**: allethrin-exposed rats +100 mg/Kg BW of *Rhodomyrtus tomentosa*, **(A3)**: allethrin-exposed rats +200 mg/Kg BW of *Rhodomyrtus tomentosa*, **(A4)**: allethrin-exposed rats +300 mg/Kg BW of *Rhodomyrtus tomentosa* (^ns^p >0.05, ^##^ *p* < 0.01 vs A-, *p < 0.05 vs A+, **p < 0.01 vs A+).

## 3 Discussion

In rat models subjected to allectrin-containing electric mosquito repellents, 100–300 mg/kg BW *R. tomentosa* impacted hematological parameters. Neutrophils, hematocrit, and urea were similar. Electric mosquito repellents with allectrins cause oxidative stress in model rats’ lung tissue. These modifications include more hemoglobin, leukocytes, lymphocytes, eosinophils, and monocytes (Situmorang et al., 2021a). The average diameter distribution of Haramonting is 600.1 nm ± 135.8. The LC50 and LD50 values for Haramonting are 2,961.535 ppm and 10.4 ± 0.135 mg/kg BW, respectively. Therefore, it has a low level of toxicity (Situmorang et al., 2021b). The histological examination of the heart, kidneys, lungs, and brain was conducted to assess toxicity (Situmorang et al., 2021b). The investigation revealed that a dosage of 400 mg/kgBW resulted in histological damage to these organs, So the dosage used in this trial did not exceed 300 mg per kilogram of body weight (Situmorang et al., 2021b). *Rhodomyrtus tomentosa* can control these cells because it contains antioxidants that fight free radicals (Lai et al., 2015; Zhang et al., 2018). *Rhodomyrtus tomentosa regulated* SOD, MDA, and NGAL expression at 200–300 mg/Kg BW, but the comparison group, A1 (Vitamin C), and A4 groups did not differ. Lack of antioxidants increases lipid peroxide activity, which enhances MDA and NGAL and lowers SOD. SOD deficiency increases MDA in injured tissues (Buyukokuroglu et al., 2008). If superoxide anions remain high, undetected tissue damage can ensue. Radical superoxide anions are very reactive (Phaniendra et al., 2015). Haramonting’s antioxidants reduce blood MDA and NGAL, increasing SOD activity. *Rhodomyrtus tomentosa* increases SOD activity, protecting cells against oxidant disturbances and oxidative stress, which can cause disease and lung tissue injury (Lavanya et al., 2012).

The article "Rhodomyrtus tomentosa (Aiton) Hassk. (haramonting) protects against allethrin-exposed pulmo damage in rats: mechanistic interleukins" was retracted in 2026. Reasons: duplicated images; unreliable data; unreliable results or conclusions.

The A+ (allethrin-exposed) group had the highest IL-1β expression, while the A- and *R. tomentosa* 300 mg/kg BW groups had the lowest. Allethrin can cause bronchitis and lung damage in asthmatics (Hernández et al., 2011). The potential hazards of alltehrin on respiratory health in mosquito coils arise due to suspicions that producers of these coils do not fully disclose all the components in their chemical analysis reports (Kasumba et al., 2016). An analysis of the organic chemistry and elemental makeup of mosquito coil ash is necessary to determine the specific compounds present in the matrix (Abdulla Al-Mamun et al., 2017). Indoor usage of mosquito repellant can result in the accumulation of substantial quantities of ash particles and toxins. Allethrin is the sole organic ingredient in mosquito repellent that has environmental and human concerns (Vorselaars et al., 2021). IL-1β is a powerful pro-inflammatory cytokine secreted after infections and traumas (Hernández et al., 2011). Allethrin, an iNOS-containing drug, reduced IL-1β levels in lung tissue using immunohistochemical examination (Indalao et al., 2017). IL-1β promotes the development of active B lymphocytes into plasma cells by promoting monocytes to become conventional dendritic cells (DCs) and macrophages (Indalao et al., 2017). Flow cytometry was used to detect cytokines at the protein level on IL-1β, a secreted isoform of IL-1β. Recent mouse studies suggest that IL-1β stimulation drives smoke-induced inflammation without inflammation (Jiang et al., 2023). *Rhodomyrtus tomentosa* antioxidants directly react with free radicals, minimizing oxidative damage. They indirectly reduce oxidative damage by lowering free radical-generating enzymes or enhancing antioxidant enzymes in cells (Zhang et al., 2018). The DPPH assay gave the methanol extract an IC50 of 107 g/mL, the FRAP assay gave it 0.162 nm at 500 g/mL, and the Metal Chelating Assay gave it 36% at 100 g/mL. HPLC showed gallic acid, tannic acid, and quercetin (Sukweenadhi et al., 2020). *Rhodomyrtus tomentosa* is utilized as an antioxidant in food to prevent oxidation (Lavanya et al., 2012; Lai et al., 2015). It is used in pharmaceuticals as an alternative antioxidant to protect biomolecules from free radical damage in a variety of human illnesses (Lavanya et al., 2012).

The article "Rhodomyrtus tomentosa (Aiton) Hassk. (haramonting) protects against allethrin-exposed pulmo damage in rats: mechanistic interleukins" was retracted in 2026. Reasons: duplicated images; unreliable data; unreliable results or conclusions.

Control (A-) and vitamin C (A1) groups expressed the greatest IL-6, whereas A4 expressed the least. Lung vitamins like vitamin C are antioxidants. It helps overcome chronic respiratory disorders. Oxidative stress from toxins and free radicals damages lung tissue, especially in chronic lung disease patients (Lei et al., 2022). Vitamin C protects alveoli and reduces COPD risk (Lei et al., 2022). We employed Vitamin C as a control due to its previous utilization in lung health research as a preventive measure and an anti-inflammatory agent (Hemilä and Douglas, 1999; Chambial et al., 2013; Holford et al., 2020). Allethrin induces IL-6 expression by stimulating the infiltration of myeloid-derived suppressor cells, neutrophils, and inflammatory stem-like cells via Janus-activated signal transducers/kinases and transcription pathway 3 activators (Ibrahim et al., 2020). These cytokines reduce inflammation (Ibrahim et al., 2020). *Rhodomyrtus tomentosa* leaf extract is antioxidant-rich. Antioxidants prevent oxidation by transforming reactive free radicals into stable ones. Mouse studies show that mitochondrial antioxidants prevent inflammation and organ failure (Zhang et al., 2018). IL-6 receptor signaling reduces oxidative stress and allethrin-induced damage (Qing et al., 2020). IL-8 expression was highest in allethrin-exposed groups and lowest in *R. tomentosa* 300 mg/kg BW (A4) groups. Allethrin attacks neutrophils and other immune cells at the infection site, causing inflammation and IL-8 production. Epithelial, airway smooth muscle, and endothelial cells generate IL-8 (Pease and Sabroe, 2002). Even at low doses, IL-8 chemotaxis stimulates neutrophils to release lysosomal enzymes, upregulate adhesion molecules, increase intracellular calcium, and increase oxidative stress, which maintains *R. tomentosa* expression. Certain leukocytes and endothelial cells emit IL-8. Hypoxia and chemotherapeutic medications can also cause fibroblasts and cancer cells to release IL-8 (Gonzalez-Aparicio and Alfaro, 2020). When given to treat chronic pulmonary diseases, vitamin C reduced its expression as an antioxidant. In chronic lung disease patients, toxins and free radicals cause oxidative stress and lung tissue destruction. A quantitative UV-Vis spectrophotometer study found that the methanol fraction of *Rhodomyrtus toementosa* leaf methanol extract had the strongest antioxidant activity with an IC50 value of 51.95 g/mL (Idris et al., 2022). Inflammation-induced oxidative stress may be caused by high IL-8 and insufficient glutathione. In other words, reactive oxygen species boost interleukin-8 and decrease glutathione (Cesta et al., 2022). Thus, interleukin-8 and the oxidant-antioxidant system are linked (Cesta et al., 2022). In contrast, the control and Vitamin C (A1) groups expressed the least IL-9. Due to its immunopathological connection with T helper 2 (TH2), allethrin increased IL-9 expression in rats (Li et al., 2017). Th9 cells, which express IL-9, are overrepresented in blood and CD4^+^ T cells. Both mast cells and eosinophils, IL-9’s targets, contribute to allergic disease by releasing pro-inflammatory chemicals at inflammation sites (Li et al., 2017). IL-9, a pleiotropic cytokine, can cause allergic inflammation and cause eosinophilic inflammation, mucosal gland hyperplasia and hypertrophy, and bronchial hyperreactivity in asthmatics (Li et al., 2022). Vitamin C’s anti-inflammatory, immune-supportive, and cofactor role for mono- and dioxygenases may have reduced IL-9 expression after supplementation (Ellulu et al., 2015). Water-soluble vitamin C protects cells inside and out from free radical damage. Vitamin C helps free radicals stabilize by providing electrons (Lobo et al., 2010). The antioxidant-rich herb haramonting neutralizes free radicals that damage lung tissue. Free radical damage can cause lung cancer and other issues. Our bodies produce some antioxidants, but Haramonting must be obtained from diet or herbal supplements.

The article "Rhodomyrtus tomentosa (Aiton) Hassk. (haramonting) protects against allethrin-exposed pulmo damage in rats: mechanistic interleukins" was retracted in 2026. Reasons: duplicated images; unreliable data; unreliable results or conclusions.

IL-10 expression was highest in the control (A-) and vitamin C (A1) groups and lowest in the A+ group. Allethrin-exposed rats have low levels of IL-10, which selectively blocks the CD28 co-stimulatory pathway in T cells to inhibit and develop antigen-specific immunity (Dennis et al., 2013). IL-10 only suppresses T cells triggered by a few activated T cell receptors, hence CD28 costimulation is needed (Dennis et al., 2013). IL-10 controls innate and cell-mediated immunity and homeostasis (Iyer and Cheng, 2012). IL-10 inhibits cell cytokine, activated antigen, and mitogen production. Free radical damage from allethrin, mutagens, and stimulants like neutrophils and monocytes is prevented by vitamin C (Rojas et al., 2017). Super Oxide Dismutase (SOD) converts oxygen to hydrogen peroxide. Zinc enhances the hydroxyl radical (OH)-removing chemical metallothionein (Marreiro et al., 2017). Vitamin C increases natural killer cell activity and lymphocyte expansion (Carr and Maggini, 2017). Terpenoids and steroids in *R. tomentosa* have significant antioxidant properties, with IC50 values of 6–50 ppm (Hamid et al., 2017). Rhodomyrtus tomentosa 300 mg/kg BW (A4) and A-expressed the least IL-18, while A+ expressed the most. A+ cells produce more IL-18 because it activates Th1 cells and increases FasL, which promotes CD8^+^ T and NK cell cytotoxicity (Widowati et al., 2020). IFN- production is another inflammatory cytokine boosted by IL-18. IL-18, like IL-1, is produced by macrophages, dendritic cells, possibly lymphocytes, and nonimmune cells. Its function is regulated by the expression of its receptors by a variety of targets, proteinase cleavage, and blocking proteins. Since monocytes, macrophages, keratinocytes, and mesenchymal cells produce IL-18, a dose of 100 mg/kgBW is appropriate. *Rhodomyrtus tomentosa’s* IL-18 suppression is insufficient. The superiority of A1 over A3 is not always apparent, suggesting that this plant may have advantages over Vitamin C. Perhaps, it could become an antioxidant-rich medicinal ingredient in the future. This is strengthened by its phytochemicals and antioxidants. Rhodomyrtone, a primary plant-derived component from *R. tomentosa* (Myrtaceae) leaf extract, may be a natural antioxidant (Wunnoo et al., 2021). The plant’s herbal component reduced IL-18 expression at 200–300 mg/kg body weight. LPS decreased RAW cell NO production with IC50 values of 3.8–74.3 M (Vo and Ngo, 2019). The phloroglucinol derivative from *R. tomentosa* leaves had anti-inflammatory properties (Vo and Ngo, 2019). Another intriguing study found that *R. tomentosa* controls immune system gene expression to reduce inflammation. Kidney head macrophages showed elevated IL-1β, IL-8, and TNF□β levels, while IL-10 and TGFβ expression was boosted (Kany et al., 2019). Rhodomyrtone inhibits the NF-B, ERK, JNK, and p38 signaling pathways to promote cutaneous organ cultures by decreasing TNF- and IL-17A transcription and expression (Wunnoo et al., 2021). Rhodomyrtone also inhibits keratinocyte hyperproliferation, treating various inflammatory cytokine-mediated diseases (Wunnoo et al., 2021).

The article "Rhodomyrtus tomentosa (Aiton) Hassk. (haramonting) protects against allethrin-exposed pulmo damage in rats: mechanistic interleukins" was retracted in 2026. Reasons: duplicated images; unreliable data; unreliable results or conclusions.

## 4 Conclusion

In Conclusion, the concentrations of pro-inflammatory cytokines IL-1β, IL-8, IL-9, and IL-18 are elevated in both the bloodstream and tissues after being exposed to an electric mosquito repellent that contains allethrin. Nevertheless, the concentrations of anti-inflammatory cytokines IL-6 and IL-10 are reduced. Allethrin stimulates the production of reactive oxygen species (ROS), which leads to the alteration of the antioxidant response in this plant through the involvement of IL-6, IL-10 in Haramonting administration, and Vitamin C. The connection between autophagy and the antioxidant response will be established by IL-6 and IL-10, resulting in a reduction of reactive oxygen species (ROS) in the lungs. This reduction will result in an elevation of the crucial antioxidant factor NRF2, which will rapidly migrate to the mitochondria to suppress mitochondrial function and stimulate mitophagy. Moreover, it is probable that cellular levels of cyclic adenosine monophosphate (cAMP) play a role in promoting mitophagy, which is the process of removing damaged mitochondria, in order to decrease the production of reactive oxygen species (ROS). *Rhodomyrtus tomentosa* has the potential to enhance alveolar histological changes. Similar to the Vitamin C group, it reduces the expression of IL-1β, IL-8, IL-9, and IL-18, while increasing the expression of IL-6 and IL-10. The administration of Haramonting results in a substantial increase in the levels of IL-6 and IL-10. This study provides Supplementary Material on the association between the effectiveness of a medicinal plant and the synthesis of cytokines.

## Data Availability

The original contributions presented in the study are included in the article/Supplementary Material, further inquiries can be directed to the corresponding author.
